RETRACTED

# IMP3 accelerates the progression of prostate cancer through inhibiting PTEN expression in a SMURF1-dependent way

**DOI:** 10.1186/s13046-020-01657-0

**Published:** 2020-09-16

**Authors:** Xiang Zhang, Dawei Wang, Boke Liu, Xingwei Jin, Xianjin Wang, Junwei Pan, Weichao Tu, Yuan Shao

**Affiliations:** 1 Department of Urology, Ruijin Hospital, Shanghai Jiaotong University School of Medicine, No. 197, 2nd Ruijin Road, Shanghai, 200025 PR China; 2 Department of Urology, Ruijin Hospital North, Shanghai Jiaotong University School of Medicine, No. 999, Xiwang Road, Shanghai, 201801 China

**Keywords:** Prostate cancer, IMP3, PTEN, PI3K/AKT/mTOR, SMURF1, Ubiquitination

## Abstract

**Background:**

Insulin-like growth factor 2 (IGF2) messenger RNA binding protein 3 (IMP3) has been testified to be overexpressed in prostate cancer and strongly related to patients’ poor prognosis. However, the functions of IMP3 and the underlying mechanisms in prostate cancer still remain unknown. Therefore, the current study was carried out to reveal the role and molecular mechanism of IMP3 in prostate cancer progression.

**Methods:**

The expression levels of IMP3 in prostate cancer tissues and cells were detected by immunohistochemistry (IHC), western blotting and RT-PCR. CCK-8, clone formation, flow cytometry and in vivo tumor formation assays were used to determine cell growth, clone formation apoptosis and tumorigenesis, respectively. The effect of IMP3 on the expression levels of the key proteins in PI3K/AKT/mTOR signaling pathway, including PIP2, PIP3, p-AKT, AKT, p-mTOR, mTOR, PTEN and BAD activation of was determined by western blotting. IP (Immunoprecipitation) assay was used to evaluate the effects of IMP3 and SMURF1 (SMAD specific E3 ubiquitin protein ligase 1) on the ubiquitination of PTEN protein.

**Results:**

IMP3 expression level was significantly increased in prostate cancer tissues and cell lines (LNCap, PC3 and DU145) as compared with the paracancerous normal tissues and cells (RWPE-1), respectively. High expression of IMP3 apparently promoted cell viability, tumorigenesis and inhibited cell apoptosis in prostate cancer LNCap, DU145 and PC3 cell lines. In mechanism, IMP3 upregulation significantly increased the phosphorylation levels of AKT and mTOR, and elevated PIP3 expression level, while induced significant reductions in the expression levels of BAD, PTEN and PIP2. And, IMP3 overexpression increased SMURF1 expression, which facilitated PTEN ubiquitination. In addition, SMURF1 overexpression enhanced prostate cancer cell viability and inhibited cell apoptosis. Silence of SMURF1 rescued the enhancements in cell proliferation and tumorigenesis and the inhibition in cell apoptosis rates induced by IMP3 in prostate cancer DU145 and LNCap cells.

RETRACTED

**Conclusion:**

This study reveals that IMP3 is overdressed in prostate cancer, which accelerates the progression of prostate cancer through activating PI3K/AKT/mTOR signaling pathway via increasing SMURF1-mediated PTEN ubiquitination.

## Background

Prostate cancer is the second common malignancy in US, with 174,650 new cases and 31,620 deaths in 2019 [1]. Ethnicity, age, family history and genetics have been identified as the risk factors of prostate cancer [2]. Although big processes having been achieved in the treatment options, such as surgery, external beam radiation therapy, brachytherapy and the combination of radiotherapy with androgen deprivation therapy [3], prostate cancer still remains the third most common reason for cancer-related death in men [4, 5]. Therefore, it is essential to further expound the mechanisms underlying this disease.

Insulin-like growth factor 2 (IGF2) messenger RNA binding protein 3 (IMP3), also known as IGF2BP3, is one of the three members of IGF2BP family which modulates the transport and translation of mRNA though binding to the coding regions of target mRNAs, such as IGF2, MYC, and β-actin [6–8]. IMP3 has been identified as an oncofetal protein, which is overexpressed and predicts a poor prognosis in several kinds of human cancers, such as breast cancer [9], cervical cancer [10], colon cancer [11] and bladder cancer [12]. Studies also demonstrated that IMP3 serves as an oncogene in carcinogenesis. For instance, Bhargava et al. [13] demonstrated that IMP3 promoted glioma cell migration through increasing the translation of RELA/p65. Pasiliao et al. [14] reported that IMP3 facilitated cell migration, invasion, and adhesion in pancreatic cancer. In prostate cancer, IMP3 level is significantly elevated in the tissue and serum samples of prostate cancer patients, which correlates with higher Gleason scores and poor cancer-specific survival [15–17]. However, the functions and mechanisms of IMP3 in prostate cancer progression still remain largely unknown.

The PI3K/AKT/mTOR signaling has been reported to be hyperactivated in multiple kinds of cancers, including prostate cancer, leading to cell growth promotion and apoptosis repression [18, 19]. PTEN (phosphatase and tensin homolog), located in human chromosome 10q23.3, is a negative regulator of PI3K/AKT/mTOR signaling [20]. Notably, PTEN has been identified as one of the most frequently deleted tumor suppressor genes in prostate cancer [21, 22], which significantly contributes to the malignant progression of prostate cancer [23–25]. It has been recently reported that PTEN can be modulated via posttranslational modifications, such as ubiquitination [26]. IMP3 has been demonstrated to downregulate the expression of p53, which is a downstream factor of PTEN/PI3K/AKT signaling [27], hence we conjecture that IMP3 might modulate the activation of PTEN/PI3K/AKT signaling.

RETRACTED

In the current study, we aimed to disclose IMP3 roles in the progression of prostate cancer, as well as to determine whether IMP3 can modulate the PTEN/PI3K/AKT/mTOR signaling.

## Materials and methods

### Tissue samples

Twenty paired prostate cancer tissues and the adjacent normal tissues were obtained from prostate cancer patients who received radical prostatectomy between August 2016 and October 2018. Among these 20 patients, 8 patients were diagnosed with organ-confined carcinomas and 7 cases were present with metastatic prostate cancer and 5 cases were diagnosed with castration-resistant prostate cancer. All patients signed the informed consent prior to this study. Experiments involving human samples have been performed referring to the Helsinki Declaration and were approved by the ethical committee of Ruijin Hospital North, Shanghai Jiao Tong University.

### Immunohistochemistry (IHC)

The expression of IMP3 in human prostate tissues and the adjacent normal tissues were immunohistochemically evaluated using anti-IMP3 antibody (No. ab179807, Abcam, MA, USA) at 1:250 dilution with a 3-step immunoperoxidase technique. In brief, the tissues were deparaffinized, hydrated, immersed in citrate buffer and autoclaved followed by incubation with rabbit serum for 30 min. Following incubation with the primary antibody for 24 h at 4 °C, the slides were washed with PBS and incubated with the corresponding secondary antibodies. Chromogen 3, 3′-diaminobenzidine tetrachloride (DAB) (Serva, Heidelberg, Germany) was used as a substrate. Cell nucleus was stained with Harri’s hematoxylin solution (Solarbio, Beijing, China). Two experienced pathologists who blinded to the clinical data, evaluated IMP3 staining based on the percentage of positive and intensity of IMP3 staining [28]. Stained area in each region of interest: 0 for a percentage < 5%, 1 for 5–25%, 2 for 25–50%, 3 for 50–75%, and 4 for > 75%. The intensity of staining was scored as 0, 1, 2 and 3 for the representation of negative (no staining), mild (weak but detectable above control), moderate (distinct) and intense (strong). The percentage of positively stained area and intensity of staining were multiplied to produce a weighted score.

### Cell line and culture condition

One human normal epithelial prostate cell line RWPE-1, and three prostate cancer cell lines PC3, LNCap and DU145, were purchased from American Type Culture Collection (ATCC, Manassas, VA, USA). RWPE-1 and DU145 cells were grown in Dulbecco’s Modified Eagle Medium (DMEM), LNCap cells were cultured in Roswell Park Memorial Institute-1640 (RPMI-1640) medium and PC3 cells were cultured in F-12 K medium, with 10% FBS and 1% penicillin/streptomycin supplementation. All cells were maintained in humidified air at 37 °C with 5% CO_2_. Dulbecco’s modified eagle medium (DMEM), F-12 K medium, Roswell Park Memorial Institute-1640 (RPMI-1640) (1X), and fetal bovine serum (FBS), and penicillin/streptomycin were purchased from Thermo Fisher Scientific (MA, USA).

RETRACTED

In addition, cells were treated with 100 mg/ml cycloheximide (CHX, Solarbio) to inhibit protein synthesis. MG132 (10 μg/ml; MCE, NJ 08852, USA), a proteasome inhibitor was used to inhibit proteasome in prostate cancer cells.

### Constructs of lentivirus vectors and transfections

Small interfering RNAs (siRNAs) used to silence IMP3 (si-IMP3), the overexpressing lentivirus vectors, OE-IMP3 and OE-SMURF1 (SMAD specific E3 ubiquitin protein ligase 1), together with the short hairpin RNA (shRNA) of SMURF1 (sh-SMURF1) and the negative control vectors (NC) all were obtained from GenePharma Co., LTD (Shanghai, China). The vectors of si-IMP3 and si-NC were transfected into prostate cancer cells with the help of Lipofectamine 2000 reagent (Invitrogen, California, USA) according to the manufactory’s descriptions. The lentivirus vectors, including OE-IMP3, OE-SMURF1, shRNA-SMURF1, OE-NC and sh-NC were introduced into cells by cell infection technology with the help of 7 μg/ml polybrene. The infected cells were selected with 7 μg/ml puromycin and/or 100 μg/ml G418 for 14 days to construct the stale transfection cells if necessary.

### RNA isolation and real-time PCR (RT-PCR)

Total RNA was isolated from tissues and cells using RNAeasy RNA isolation kit (Qiagen, Valencia, CA, USA) according to the manufactory’s instructions. After being quantitated using a NanoDrop ND 1000 Spectrophotometer (NanoDrop Technologies Inc., Wilmington, DE, USA), a total of 1 μg RNA was transformed into cDNA through reverse transcription using First Strand cDNA Synthesis Kit for RT-PCR (Roche, Indianapolis, IN, USA). RT-PCR was performed on a Roche Light cycler 480 Real-Time PCR System using SYBR green master mix (Thermo Fisher Scientific, MA, USA). Gene expressions were normalized to the level of GAPDH and calculated by 2^-ΔΔCt^ method [29]. Specific primers were designed and synthesized by Invitrogen and were listed in Table 1.

**Table 1:** Primer sequences used in RT-PCR

Gene	Forward (5′-3′)	Reverse (5′-3′)
IMP3	TCGGAAACCTCAGCGAGAAC	ACTATCCAGCACCTCCCACT
SMURF1	GCTTCAAGGCTTTGCAAGGTT	TGGGAGCCACCAACAAAAGT
GAPDH	CCACTAGGCGCTCACTGTTCT	GCATCGCCCCACTTGATTTT

RETRACTED

### Western blotting analysis

Total proteins were isolated from cells and tissues using RIPA buffer (50 mM Tris-HCL, 150 mM NaCl, 0.1% SDS, 1% NP40 and 0.5% sodium deoxycholate) supplemented with 1% protease inhibitor (Solarbio). The lysate was thawed in ice, and the cellular lysates were mechanically disrupted by scrape through tips and the supernatants were collected after centrifugation at 13, 000 rpm for 30 min at 4 °C. Following concentrations being determined using a Bio-Rad DC Protein Assay kit (Thermo Fisher Scientific), 30 μg proteins from each sample were loaded on a 10% PAGE gel and then transferred onto the polyvinylidene fluoride membranes (Millipore, Billerica, MA, USA). Subsequently, the membranes were probed with the indicated primary antibodies, including IMP3 (No. ab179807, Abcam), PIP2 (No. sc-53,412, Santa Cruz Biotechnology, Dallas, Tx, USA), PIP3 (No. AV46228, Sigma-Aldrich, MO, USA), p-AKT (No. ab38449, Abcam), AKT (No. ab18785, Abcam), PTEN (No. ab32199, Abcam), p-mTOR (No. ab109268, Abcam), mTOR (No. ab2732,Abcam), BAD (No. ab32445, Abcam), Ub (No. ab7780, Abcam), SMURF1 (No. ab57573, Abcam), CDC4 (No. ab74054, Abcam), RCHY1 (No. ab189907, Abcam), MDM2 (No. ab38618, Abcam), SKP2 (No. ab68455, Abcam), UBE3A (No. ab126765, Abcam), GAPDH (No. ab181602, Abcam) overnight at 4 °C, followed by incubation with the corresponding HRP-conjugated secondary antibodies (Santa Cluz Biotechnology). Signals were enhanced with ECL reagent (Millipore) and imaged on a gel imaging system (Odyssey, LI-COR Biosciences).

### Immunoprecipitation (IP) assay

The interaction between PTEN and Ub proteins was evaluated by IP assay. In brief, prostate cancer cells were washed with cold PBS and then lysed with IP lysis buffer (Thermo Fisher Scientific). Subsequently, cell lysate containing 200 μg proteins was incubated with Dynabeads® protein G for 1 h at room temperature, and cross-linked with 2 μg of antibody against PTEN (No. ab32199, Abcam) or Ub (No. 3936, Cell Signaling Technology, MA, USA) overnight at 4 °C. Next, the proteins were incubated with Dynabeads® protein G for another 1 h to form the immune complex which was loaded onto gels using anti-Ub (No. 3936, Cell Signaling Technology) or anti-PTEN (No. ab32199, Abcam) antibody.

### CCK-8 assay

Cell Counting Kit-8 kits (Dojindo, Japan) were applied to assess prostate cancer cell proliferation ability. In briefly, cells were seeded into 96-well plates at a density of 2 × 10^3^ cells per well and incubated at 37 °C overnight, followed by cell transfections or infections. After 1, 2, 3, 4, or 5 days of cell incubation at 37 °C, 10 μL of CCK-8 solution was added into each well of the 96-well plates and the cells were incubated at 37 °C for another 4 h. Absorbance at 450 nm was measured under a Microplate Reader (Bio-Rad, Hercules, CA, USA).

RETRACTED

### Cloning formation assay

The stably transfected prostate cell lines were trypsinized and inoculated into 6-well plates at a density of 2000 cells/100 μL each well and incubated at 37 °C for 14 days, with medium replacement every 2 days. After that, the medium was removed and the cells were washed with PBS twice, following by being fixed with 5% paraformaldehyde for 30 min. Then, the cells were incubated with 0.1% crystal violet solution (Solarbio) for 20 min at room temperature. The visible colonies were counted under microscope.

### Flow cytometry

Prostate cancer cells transfected with si-IMP3, si-NC or infected with OE-IMP3, OE-NC, OE-SMURF1, sh-SMURF1 or OE-IMP3 + sh-SMURF1 were trypsinized and washed in ice-cold PBS. Subsequently, the cells were incubated with Annexin V-FITC/propidium solution (BD Bioscience, San Diego, CA, USA) prior to flow cytometric analysis. Stained cells were assayed in a fluorescence-activated cell sorter (Becton Dickinson, Franklin Lakes, NJ, USA) and the apoptotic cells were analyzed by using Flowjo 7.6 software.

### Tumor formation experiment

Animal assay was performed in accordance to the institutional guidelines and approved by the Experimental Animal Center of Ruijin Hospital North Shanghai Jiao Tong University School of Medicine. Four-week-old male BALB/c-nude mice were used for the in vivo assay. First, a total of 1 × 10^6^ PC3 and LNCap cells stably transfected with OE-IMP3 or OE-IMP3 + sh-SMURF1 were subcutaneously injected into the armpit area of mice. At 28 days post-injection, the tumors were taken out and weighted.

### Statistical analysis

Statistic Package for Social Science (SPSS) 22.0 statistical software (IBM, Armonk, NY, USA) was used for data analysis. Picture was edited using GraphPad Prism 5.0 software (Version X; La Jolla, CA, USA). Data are presented as mean ± standard deviation (mean ± SD) and the comparisons between 2 groups and multiple groups (≥3 groups) were executed using t tests and One-way ANOVA followed by Dunnett’s post-hoc tests, respectively. *p* < 0.05 was considered as statistically significant. ^*, #^ *p* < 0.05, ^**, ##^ *p* < 0.01 and ^***, ###^ *p* < 0.001.

## Results

### IMP3 is highly expressed in prostate cancer tissues and cell lines

To explore the roles and molecular mechanisms of IMP3 in prostate cancer, we first assessed the expression profiles of IMP3 in prostate cancer tissues and cell lines. As detected by the RT-PCR, western blotting and IHC technologies, significant increases in IMP3 mRNA and protein levels were observed in prostate cancer tissues as compared with the normal tissues (Fig. 1a-c). Similarly, the mRNA and protein levels of IMP3 in prostate cancer cell lines, including LNCap, PC3 and DU145 were obviously higher than those in the normal prostate epithelial cell line RWPE-1 (Fig. 1d-e). These results suggested that IMP3 was overexpressed in prostate cancer tissues and cells.

RETRACTED

**Fig. 1:** IMP3 expression was elevated in prostate cancer tissues and cells. **a**-**b** RT-PCR and western blotting assays were performed to examine the mRNA and protein expression levels of IMP3 in 20 paired prostate cancer tissues and normal tissues, the representative blots were shown in (**c**). IHC technology was carried out to test IMP3 protein levels in prostate cancer tissues and the matched normal tissues with anti-IMP3 antibody, and the representative images of each group were shown in (**d**-**e**). RT-PCR and western blotting assays were performed to examine the mRNA and protein expression levels of IMP3 in RWPE-1, LNCap, PC3 and DU145 cell lines. (^**^p < 0.01, ^***^p < 0.001, compared with normal/RWPE-1 group)

### IMP3 functions as an oncogene in prostate cancer

Then, we performed the gain- and loss-of-function assays to evaluate IMP3 roles in the progression of prostate cancer. Compared with si-NC group, the expression of IMP3 was significantly reduced after DU145, LNCap and PC3 cells were transfected with si-IMP3–1 at both mRNA (Fig. 2a) and protein levels (Fig. 2b). Meanwhile, OE-IMP3 induced a notable increase in IMP3 expression (Fig. 2a-b). As si-1 presented with the highest knockdown efficiency among the 3 siRNAs targeting IMP3 gene, si-1 was selected for further study. Overexpression of IMP3 in PC, DU145 and LNCap cells led to obvious enhancements in cell proliferation (Fig. 2c-e) and clone formation abilities (Fig. 2f), while inhibited cell apoptosis (Fig. 2g-h). On the contrary, silence of IMP3 repressed cell proliferation (Fig. 2c-e) and clone formation abilities (Fig. 2f) and induced cell apoptosis (Fig. 2g-h). These results demonstrated that IMP3 served as an oncogene in prostate cancer progression.

**Fig. 2:** Overexpression of IMP3 promoted prostate cancer cell proliferation and repressed cell apoptosis. **a**-**b** The mRNA and protein expression levels of IMP3 in PC3, LNCap and DU145 cells of si-NC, si-IMP3, OE-NC and OE-IMP3 groups were determined by using RT-PCR and western blotting assays, respectively. **c**-**e** Cell proliferation ability was determined by CCK-8 assay in different groups of PC3, LNCap and DU145 cells, including si-IMP3, si-NC, OE-IMP3 or OE-NC groups. **f** Cell clone formation ability was tested by clone formation assay after PC3, LNCap and DU145 cells were transfected with si-IMP3, si-NC, OE-IMP3 or OE-NC. **g**-**h** The apoptosis rates of PC3, LNCap and DU145 cells in si-IMP3, si-NC, OE-IMP3 or OE-NC groups were tested by flow cytometry assay (Cells in Q2 and Q3 were considered as the apoptotic cells). (^*^p < 0.05, ^***^p < 0.001, si-IMP3 group compared with si-NC group; ^#^*p* < 0.05, ^##^*p* < 0.01, ^###^*p* < 0.001, OE-IMP3 group compared with OE-NC group)

RETRACTED

### IMP3 activates PI3K/AKT/mTOR signaling via increasing PTEN ubiquitination in DU145 and LNCap cells

Then, IMP3 role in the activation of PI3K/AKT/mTOR pathway in prostate cancer cells was explored. Compared with the OE-NC group, upregulation of IMP3 obviously increased the expression levels of PIP3, p-AKT and p-mTOR, while reduced the expression levels of PIP2 and BAD in PTEN-null PC3 cells (Fig. 3a), together with a decrease in PTEN expression in DU145 and LNCap cells (Fig. 3b-c). In addition, we observed that overexpression of IMP3 induced a significant decrease in PTEN protein stability in LNCap and DU145 cells (Fig. 3d-f), and promoted PTEN degradation via ubiquitination pathway (Fig. 3g-n). These results suggested that IMP3 overexpression decreased PTEN expression in DU145 and LNCap cells, leading to the activation of PI3K/AKT/mTOR signaling.

**Fig. 3:** IMP3 promoted the activation of PI3K/AKT/mTOR signaling and facilitated the ubiquitination of PTEN protein in prostate cancer cells. **a**-**c**. The expression levels of PIP2, PIP3, p-AKT, AKT, p-mTOR, mTOR, PTEN and BAD were determined by western blotting technology after IMP3 were upregulated or downregulated in PC3, LNCap and DU145 cells. **d**-**f**. Following cell transfection/infection with si-IMP3, si-NC, OE-IMP3 or OE-NC for 24 h, DU145 and LNCap cells were treated with 100 μg/ml of CHX for 0, 1, 2, 4, 8 or 24 h, then total proteins were extracted from cells and submitted to western blotting to detect the expression of PTEN protein. **g**-**i**. The ubiquitination level of PTEN protein was determined by IP assay after cell transfection/infection with si-IMP3, si-NC, OE-IMP3 or OE-NC in DU145 and LNCap cells with anti-PTEN antibody. **j**-**l**. The ubiquitination level of PTEN protein was determined by IP assay with anti-Ub antibody. **m**-**n**. The ubiquitination level of PTEN protein was determined by IP assay after cell treatment with MG132 (10 μg/ml) for 4 h or without. (^*^p < 0.05, ^**^p < 0.01, si-IMP3 group compared with si-NC group; ^#^*p* < 0.05, ^##^*p* < 0.01, OE-IMP3 group compared with OE-NC group)

### IMP3 increases SMURF1 expression

Then, we explored the mechanism by which IMP3 promoted the ubiquitination of PTEN protein in DU145 and LNCap cells. Compared with control group, upregulation of IMP3 significantly increased the protein expression level of SMURF1, with no obvious influence in the expression levels of other ubiquitination-related proteins, such as CDC4, URB5, RCHY1, MDM2, SKP2 and UBE3A in DU145 (Fig. 4a) and LNCap cell lines (Fig. 4b). To further assess the relationship between SMURF1 and IMP3, RT-PCR was carried out. As shown in Fig. 4c-d, IMP3 overexpression significantly increased SMURF1 mRNA level in DU145 and LNCap cells, and vice versa. These results demonstrated that SMURF1 might be involved in IMP3-induced ubiquitination of PTEN.

RETRACTED

**Fig. 4:** IMP3 positively modulated SMURF1 expression in DU145 and LNCap cells. **a**-**b**. Following cell transfection/infection with si-IMP3, si-NC, OE-IMP3 or OE-NC, total RNA was isolated from cells and western blotting assay was performed to detect the protein expression levels of IMP3, CDC4, RCHY1, MDM2, SKP2, UBE3A and SMURF1. **c**-**d**. The expression of SMURF1 mRNA was determined by RT-PCR in different groups of DU145 and LNCap cells, including si-IMP3, si-NC, OE-IMP3 and OE-NC groups. (^*^p < 0.05, ^***^p < 0.001, si-IMP3 group compared with si-NC group; ^#^*p* < 0.05, ^##^*p* < 0.01, ^###^*p* < 0.001, OE-IMP3 group compared with OE-NC group)

### SMURF1 enhances the ubiquitination of PTEN protein and promotes cancer progression

To uncover SMURF1 role in IMP3-induced ubiquitination of PTEN protein, we recruited the lentiviral vectors (OE-SMURF1 and sh-SMURF1) to upregulate and silence SMURF1 in prostate cancer DU145 and LNCap cells. The mRNA and protein levels of SMURF1 were significantly elevated when the cells were infected with OE-SMURF1 as compared with the control group, whereas sh-SMURF1–3 induced an obvious reduction in SMURF1 expression (Fig. 5a-b). As sh-SMURF1–3 showed the highest knockdown efficiency among the 3 shRNAs of SMURF1, sh-1 was used in the following experiments. Ectopic expression of SMURF1 significantly enhanced the level of ubiquitinated PTEN protein and decreased its expression in DU145 and LNCap cell lines (Fig. 5c). In addition, cell proliferation was apparently enhanced (Fig. 5d-e) and apoptosis was inhibited (Fig. 5f) when SMURF1 expression was upregulated in DU145 and LNCap cells. These results suggested that SMURF1 enhanced the ubiquitination of PTEN protein and promoted cell proliferation in prostate cancer.

**Fig. 5:** SMURF1 facilitated the ubiquitination of PTEN protein and promoted cell proliferation in DU145 and LNCap cells. **a**-**b**. The mRNA and protein levels of SMURF1 were determined by RT-PCR and western blotting assays following cell infection with OE-SMURF1, OE-NC, sh-SMURF1 or sh-NC. **c** The ubiquitination of PTEN protein was assessed by IP assay after 48 h of cell infection with OE-SMURF1, OE-NC, sh-SMURF1 or sh-NC. **d**-**e** The effects of SMURF1 up−/downregulation on cell proliferation were assessed by CCK-8 assay in DU145 and LNCap cells. **f** The effects of SMURF1 up−/downregulation on DU145 and LNCap cell apoptosis was detected by flow cytometry assay (Cells in Q2 and Q3 were considered as the apoptotic cells). (^**^p < 0.01, ^***^p < 0.001, sh-SMURF1 group compared with sh-NC group; ^#^*p* < 0.05, ^##^*p* < 0.01, ^###^*p* < 0.001, OE-SMURF1 group compared with OE-NC group)

RETRACTED

### IMP3 facilitates the progression of prostate cancer through SMURF1-mediated PTEN ubiquitination

Moreover, we investigated SMURF1 role in IMP3-mediated prostate cancer progression. Downregulation of SMURF1 rescued the increase in the ubiquitination level of PTEN induced by IMP3 overexpression in DU145 and LNCap cells (Fig. 6a), suggesting that IMP3 negatively modulated PTEN expression via promoting SMURF1-mediated PTEN ubiquitination. To reveal SMURF1 roles in IMP3-induced prostate cancer progression, CCK-8, flow cytometry and the in vivo tumor formation assays were carried out. We observed that cell proliferation enhancement and apoptosis suppression induced by IMP3 overexpression all were significantly reversed when SMURF1 was silenced in DU145 and LNCap cells (Fig. 6b-e). Furthermore, IMP3 overexpression significantly promoted the in vivo tumor formation ability of DU145 and LNCap cells, whereas this effect was abrogated by sh-SMURF1 (Fig. 6f). These results demonstrated that IMP3 facilitated the progression of prostate cancer through increasing SMURF1-mediated PTEN ubiquitination.

**Fig. 6:** IMP3 facilitated prostate cancer cell proliferation and tumorigenesis through upregulating SMURF1 expression. DU145 and LNCap cells in OE-IMP3, OE-IMP3 + sh-SMURF1 and control (OE-NC + sh-NC) groups were collected for the following assays. **a** IP assay was used to assess the crosstalk between Ub and PTEN proteins. **b**-**c** CCK-8 was applied to determine cell proliferation. **d**-**e** Flow cytometry was applied to detect cell apoptosis (Cells in Q2 and Q3 were considered as the apoptotic cells). **f** In vivo tumor formation assay was performed to detect the effect of IMP3/SMURF1 axis on the tumorigenesis of DU145 and LNCap cells. (^*^p < 0.05, ^**^p < 0.01, ^***^p < 0.001, OE-IMP3 group compared with control group; ^#^*p* < 0.05, ^##^*p* < 0.01, OE-IMP3 + sh-SMURF1 group compared with OE-IMP3 group)

## Discussion

Although the etiopathogenesis of prostate cancer is not completely clear, it is strongly postulated that gene deregulation plays a role. It has been reported that IGF family plays a key role in the angiogenesis, bone metastasis, and androgen-independent progression of prostate cancer [30]. Szarvas et al. [15] found that IMP3, a member of IMP family was positively expressed in 15% (15/101) of clinically localized prostate cancer tissues and 65% (15/23) of palliatively treated metastatic prostate cancer tissues, whereas was not detected in the benign prostate hyperplasia tissues. Similarly, Ikenberg et al. [16] also found that IMP3 was significantly overexpressed in prostate carcinomas (from a total of 476 prostate cancer tissues which includes 425 primary carcinomas and 51 prostate cancer metastases or castration-resistant prostate cancers) as compared to the normal prostate tissues. Consistently, significant increases in the mRNA and protein levels of IMP3 were observed in prostate cancer tissues and cell lines (LNCap, DU145 and PC3) as compared with normal tissues and cells.

RETRACTED

Increasing evidence has demonstrated that IMP3 plays an oncogenic role in cancers. For instance, IMP3 promoted the tumorigenesis via attenuating p53 stability in lung cancer [27]. IMP3 facilitate the metastasis and stem-like properties of triple-negative breast cancer via destabilization of progesterone receptor and regulating SLUG [31, 32]. The in vitro experiments indicated that IMP3 promoted the proliferation, motility and invasive potentials of ovarian cancer cells [33]. In the present study, we explored IMP3 roles in the progression of prostate cancer via performing the gain- and loss-of-function assays. We observed that IMP3 upregulation significantly promoted cell proliferation, clone formation viability and tumorigenesis and inhibited cell apoptosis in prostate cancer DU145, LNCap and PC3 cells. These results suggested that IMP3 served as an oncogene in prostate cancer, which was further confirmed by the loss-of-function assays induced by shRNA infection.

In mechanism, we observed that IMP3 upregulation significantly promoted the activation of PI3K/AKT/mTOR signaling in PTEN-positive DU145 and LNCap cells and PTEN-null PC3 cells. To reveal the mechanism by which IMP3 activated PI3K/AKT/mTOR signaling, we explored whether IMP3 modulated PTEN expression. The results showed that IMP3 overexpression decreased PTEN expression in DU145 and LNCap cells, while showed no affect in PTEN level in PC3 cells. We speculated that IMP3 activated PI3K/AKT/mTOR pathway through a direct manner in PC3 cells while through downregulating PTEN in LNCap and DU145 cells. Subsequently, we mainly focused on the molecular mechanism by which IMP3 induced a downregulation of PTEN level. The results showed that IMP3 overexpression accelerated the degradation of PTEN protein through increasing SMURF1-meidated PTEN ubiquitination. SMURF1 is a member of the HECT family of E3 ubiquitin ligases and was originally identified to modulate transforming growth factor-β (TGF-β)/bone morphogenetic protein (BMP) signaling via promoting the ubiquitin modification of SMADs [34]. With the development of research, other substrates of SMURF1 were identified, such as Kindlin-2 [35], Type Iγ phosphatidylinositol phosphate kinase (PIPKIγ) [36], UVRAG (UV radiation resistance associated) [37], RHOA (Ras homolog family member A) [38] and hPEM-2 (Posterior End Mark-2) [39]. Feng et al. [37] demonstrated that SMURF1 promoted the ubiquitination of UVRAG, an important regulator of mammalian macroautophagy/autophagy, resulting in autophagosome maturation and inhibition in cell growth in hepatocellular carcinoma. Here, we identified for the first time, that SMURF1 induced the ubiquitination of PTEN protein in prostate cancer DU145 and LNCap cells. We also found that knockdown of SMURF1 decreased the ubiquitylation level of PTEN induced by IMP3 upregulation, suggesting that IMP3 facilitated the ubiquitylation level of PTEN in a SMURF1-depedent manner in DU145 and LNCap cells.

RETRACTED

In addition, we found that cell proliferation was significantly enhanced and apoptosis was inhibited when SMURF1 was upregulated in prostate cancer DU145 and LNCap cells, whereas knockdown of SMURF1 inhibited cell proliferation and induced cell apoptosis. These results suggested that SMURF1 played an oncogenic role in prostate cancer, which was consistent with previous studies [40, 41]. Moreover, we observed that the oncogenic role of IMP3 in prostate cancer was abrogated when SMURF1 expression was silenced in DU145 and LNCap cells, indicating that IMP3 promoted the progression of prostate cancer via increasing SMURF1 expression.

Studies have shown that the high expression pattern of IMP3 predicted a poor prognosis in several kinds of cancers, including muscle invasive bladder cancer [12], sacral chordoma [42], hepatocellular carcinoma [43] and prostate cancer [15, 16]. However, Noske et al. [44] found that the high level of IMP3 associated with an improved survival in patients with ovarian cancer. Regrettably, we didn’t analyze the relationship between the expression levels of IMP3 and the overall survival in patients with prostate cancer mainly due to the limitation of sample size. We intend to reveal it in next studies, as well as to disclose the mechanism by which IMP3 activated PI3K/AKT/mTOR signaling in PTEN-null PC3 cells.

RETRACTED

## Conclusion

This study reveals that IMP3 accelerates the progression of prostate cancer via activating PI3K/AKT/mTOR pathway through increasing SMURF1-mediated PTEN ubiquitination. Our results demonstrated that IMP3 might be a potential target for prostate cancer treatment.

## Data Availability

All date generated or analyzed during this study were all included in this present article.

## Abbreviations

IMP3: Insulin-like growth factor 2 messenger RNA binding protein 3
PTEN: Phosphatase and tensin homolog
BMP: Bone morphogenetic protein
RHOA: Ras homolog family member A
hPEM-2: Posterior End Mark-2
